# The effects of Nigella sativa on thyroid function, serum Vascular Endothelial Growth Factor (VEGF) – 1, Nesfatin-1 and anthropometric features in patients with Hashimoto’s thyroiditis: a randomized controlled trial

**DOI:** 10.1186/s12906-016-1432-2

**Published:** 2016-11-16

**Authors:** Mahdieh Abbasalizad Farhangi, Parvin Dehghan, Siroos Tajmiri, Mehran Mesgari Abbasi

**Affiliations:** 1 Nutrition Research Center, Department of Community Nutrition, School of Nutrition, Tabriz University of Medical Sciences, Tabriz, Iran; 2 Student Research Committee, Tabriz University of Medical Sciences, Tabriz, Iran; 3 Drug Applied Research Center, Tabriz University of Medical Sciences, Tabriz, Iran

**Keywords:** Hashimoto’s thyroiditis, Nigella sativa, VEGF, Nesfatin-1

## Abstract

**Background:**

Hashimoto’s thyroiditis is an autoimmune disorder and the most common cause of hypothyroidism. The use of Nigella sativa, a potent herbal medicine, continues to increase worldwide as an alternative treatment of several chronic diseases including hyperlipidemia, hypertension and type 2 diabetes mellitus (T2DM). The aim of the current study was to evaluate the effects of Nigella sativa on thyroid function, serum Vascular Endothelial Growth Factor (VEGF) – 1, Nesfatin-1 and anthropometric features in patients with Hashimoto’s thyroiditis.

**Methods:**

Forty patients with Hashimoto’s thyroiditis, aged between 22 and 50 years old, participated in the trial and were randomly allocated into two groups of intervention and control receiving powdered Nigella sativa or placebo daily for 8 weeks. Changes in anthropometric variables, dietary intakes, thyroid status, serum VEGF and Nesfatin-1 concentrations after 8 weeks were measured.

**Results:**

Treatment with Nigella sativa significantly reduced body weight and body mass index (BMI). Serum concentrations of thyroid stimulating hormone (TSH) and anti-thyroid peroxidase (anti-TPO) antibodies decreased while serum T3 concentrations increased in Nigella sativa-treated group after 8 weeks. There was a significant reduction in serum VEGF concentrations in intervention group. None of these changes had been observed in placebo treated group. In stepwise multiple regression model, changes in waist to hip ratio (WHR) and thyroid hormones were significant predictors of changes in serum VEGF and Nesgfatin-1 values in Nigella sativa treated group (*P* < 0.05).

**Conclusions:**

Our data showed a potent beneficial effect of powdered Nigella sativa in improving thyroid status and anthropometric variables in patients with Hashimoto’s thyroiditis. Moreover, Nigella sativa significantly reduced serum VEGF concentrations in these patients. Considering observed health- promoting effect of this medicinal plant in ameliorating the disease severity, it can be regarded as a useful therapeutic approach in management of Hashimoto’s thyroiditis.

**Trial registration:**

Iranian registry of clinical trials (registration number IRCT2015021719082N4- Registered March-15-2015).

## Background

Hashimoto’s thyroiditis (HT) is an organ-specific T-cell mediated disease that affects the thyroid glands and is one of the most common human autoimmune disorders [1]. The disease affects 2% of general population and is ten times more prevalent in women than in men [2, 3]. A significant proportion of patients have asymptomatic chronic autoimmune thyroiditis and 8% of woman (10% of woman over 55 years of age) and 3% of men have subclinical hypothyroidism [4].

Hashimoto’s thyroiditis is characterized by the presence of thyroid auto-antibodies such as anti-thyroid peroxidase (TPO-Ab) and anti-thyroglobulin (TG-Ab) antibodies in the serum while these antibodies have potential ability to deteriorate thyroid cells [5, 6]. The disease is characterized by gradual thyroid failure and occasional goiter development and the untreated forms of Hashimoto’s thyroiditis can ever lead to papillary thyroid cancer and thyroid carcinoma [7, 8].

From pathological point of view, thyroid enlargement and hyper-function in Hashimoto’s thyroiditis is accompanied by a markedly increased blood flow and increased vascularization [9]. A number of growth and vasoactive factors are produced in thyroid and are considered to be potentially responsible for changes in thyroid microvasculature and blood flow; vascular endothelial growth factors (VEGF) is a hemodynamic glycoprotein with potent angiogenic and vascular permeability enhancing activities [10]. It has been proposed that VEGF and its receptors are present in epithelial cells of the thyroid and contribute in regulation of development and function of thyroid epithelial cells [10]. In fact VEGF is unique among angiogenic factors because it is both vascular endothelial cell-specific mitogen and is secreted by thyroid cancer cells and high thyroid stimulating hormone (TSH) concentrations in Hashimoto’s thyroiditis promotes VEGF secretion from thyroid cancer cell lines [11].

Nesfatin-1, a peptide secreting from peripheral tissues, central and peripheral nervous system, is involved in the regulation of energy homeostasis related with food consumption mostly by passing through the blood–brain barrier [12]. Moreover, several recent studies have proposed the possible role of Nesfatin-1 in in thyroid dysfunction [13, 14]. Liu et al. [15] reported that plasma Nesfain-1 levels are independently correlated with serum TSH concentrations in patients with T2DM. The Nesfatin-1 immuno-positive neurons have been reported to be co-localized with thyrotropin releasing hormone (TRH) neurons in the paraventricular nucleous (PVN) and the central Nesfatin-1 affects the membrane potential of TRH neurons suggesting the possible role of Nesfatin-1 in regulation of thyroid hormone function [16, 17].

Levothyroxine sodium is the treatment of choice for Hashimoto’s thyroiditis; however its chronic use is related with cardiac dysfunction, left ventricular hypertrophy [18, 19] and rapid bone loss [20]. Nigella sativa is one of the medicinal plants and belongs to the Ranunculaceae family [21]. The seeds of the Nigella sativa are the main source of its active ingredients with considerable health promoting effects including antioxidant, anti-inflammatory and immune-modulatory properties and no side effects [21, 22]. Numerous researches have extensively studied therapeutic actions of Nigella sativa in improving chronic disease status including diabetes, hyperlipidemia, hypertension and gastritis especially in animal models; while human studies in this filed are scarce and limiting [23, 24]. Moreover the health effects of Nigella sativa in Hashimoto’s thyroiditis has been studied in only one animal model indicating its protective role in reversing hypothyroid status and ameliorating oxidative stress and thyroid cell damage in propylthiouracil (PTU)-induced hypothyroidism in rats [25]. In the current randomized clinical trial we aimed to evaluate the potential therapeutic effects of Nigella sativa powder on thyroid function and serum VEGF and Nesfatin-1 concentrations in patients with Hashimoto thyroiditis.

## Methods

### Patients

In the current double-blinded placebo-controlled trial, 40 patients with Hashimoto’s thyroiditis were enrolled (Fig. 1). Subjects were recruited from outpatient endocrinology and metabolism clinics of Isfahan University of Medical Sciences. Inclusion criteria were as follows: age between 20 and 50 years and having Hashimoto’s thyroiditis according to physician diagnosis. Exclusion criteria were as follows: taking any nutritional supplements for at least 3 months prior participation or during the trial, any history of autoimmune disease, cardiovascular events, other thyroid abnormalities including Grave’s disease, being pregnant or lactating, any history of thyroid surgeries and being on any dietary regimens during and 3 months before recruitment in the trial. Participants were treated with levothyroxine while the drug dosage was stable from 6 weeks prior participation in the study to the end of the trial. The average full replacement dose of levothyroxine sodium was approximately 1.7 mcg/kg/day (e.g., 100–125 mcg/day for a 70 kg adult).

**Fig. 1:** CONSORT Flow diagram of subject recruitment

### Study design

From 100 recruited subjects, 53 participants were excluded because of not meeting the inclusion criteria or decline to participate. Among remaining 47 patients, random permuted block procedure was performed and participants were randomly allocated into Nigella sativa-treated (*n* = 23) or placebo-treated (*n* = 24) groups. During the trial, three patients in Nigella sativa-treated group were excluded from the study because of itching and nausea; while four patients in control group refused to continue the trial. Therefore, totally 20 patients in each group completed the study. Patients in the intervention group received a daily dose of 2 g Nigella sativa powder per day and placebo group received 2 g starches per day for 8 weeks. The dose of the Nigella sativa and time period of the study had been selected according to review of the previous studies indicating the effectiveness of 2 g of Nigella sativa or even lesser doses and 8 weeks study duration in treatment of numerous metabolic disorders including immune disturbances and lipid abnormalities [26, 27].

Black seed powders were obtained from corns grown in Isfahan bought by a local market (Sad-Giah market, Isfahan, Iran) and were prepared by the Goldaroo pharmaceutical company (Goldaro Pharmaceutical Co. Isfahan, Iran). The black seeds were milled in a grinder and a purified powder was prepared. The seeds were identified and authenticated by Dr. Mahdieh Abbasalizad Farhangi, supervisor of the project from Department of Nutrition, Tabriz University of Medical Sciences, Tabriz, Iran. Thereafter, Nigella sativa seeds were processed into pharmaceutical grade capsules containing Nigella sativa powder and bottled according to Good Manufacturing Practices (GMP). Each capsule was prepared containing 1 g powder of Nigella Sativa, and each bottle contained 112 capsules, for 8 weeks period of the study. While for the placebo, we used starch bought from the same market and the entire processes of its capsulation was similar to Nigella sativa seeds preparation. Participants in intervention and placebo groups received two capsules daily, taking it immediately before lunch and dinner respectively.

Randomization procedure was performed by a third investigator who had no clinical involvement in the trial to ensure complete blinding in the randomization process. Randomization was done according to computer- generated numbers and was kept in consecutively numbered envelopes opened at the moment of participant enrollment into the study. A follow-up procedure was done with weekly telephone contacts to ensure that subjects consumed the supplements regularly.

### Anthropometric and nutritional assessments

Body weight and height were measured with a calibrated digital scale and stadimeter respectively. BMI was calculated as weight (kg) divided by height (cm) squared. Waist circumference (WC) was measured in horizontal plane, midway between the lowest rib and the iliac crest with a measuring tape in centimeter. Waist to hip ratio (WHR) was calculated by WC divided by hip circumference (HC). The dietary assessments were performed using a 3-day food record, covering two weekdays and one weekend day, to estimate total energy, carbohydrate, protein, fat and antioxidant vitamins consumption. Because of the antioxidant nature of Nigella sativa the intake of vitamin E and C were specifically evaluated to ensure that no change in their consumption has been occurred throughout the trial and to rule out their possible confounding effect on study parameters. Nutrient analysis of the 3-day food record was performed using the Nutritionist IV software (N-squared Computing, Salem, OR, USA).

### Biochemical assays

Fasting blood samples were obtained from all of the participants at the beginning and end of the trial. The serum and plasma samples were separated by centrifugation at 2500 rpm for 10 min (Beckman Avanti J-25; Beckman Coulter, Brea, CA, USA) at room temperature. The serum samples were stored at −70 °C immediately after centrifugation until their assays. Serum thyroid-stimulating hormone (TSH), total triiodothyronine (T3) and total thyroxine (T4) were analyzed by enzyme linked immunosorbent assay (ELISA Kit, Pishtaz Tebe Co., Tehran, Iran) according to the manufacturer’s instructions. Anti-thyroid peroxidase antibody was measured by the commercially solid-phase ELISA kit (Aeskulisa, Wendelsheim, Germany). Serum concentration of VEGF and Nesfatin-1 were measured by commercial ELISA kits (Hangzhou East biopharm Co, USA). The sensitivity of these assays was 10.42 ng/l and 0.15 ng/ml respectively.

### Statistical assays

Statistical analysis was performed by SPSS™ statistical software (SPSS Inc., Chicago, IL, USA). Quantitative data were presented as mean ± standard deviation (SD), and qualitative data were demonstrated as frequency and percent. One-sample Kolmogorov-Smirnov test was used to assess the normality of data. Between groups comparisons of continuous variables were performed by independent sample *t*-test. Paired *t*-test was used for before and after intervention comparisons. Analysis of covariance (ANCOVA) was used to identify any differences between two treatment groups after intervention adjusting for the confounding effects of baseline concentrations of parameter, age and gender. Stepwise multivariate linear regression model was used to evaluate the predictors of changes in VEGF and Nesfatin-1 concentrations. *P*-values less than 0.05 were considered to be significant. Sample size calculation was performed based on 80% power and an α-error of 5% to detect treatment effect of Nigella sativa on serum TSH. Totally, 14 individuals were calculated. Allowing for 30% drop-out over 8 weeks of intervention, the total sample size required for the study was 40 individuals.

## Results

The flowchart of the study is given in Fig. 1. A total of 40 patients completed the study. Three patients in Nigella sativa-treated group were excluded from the study because of itching and nausea; while four patients in control group refused to continue the trial. No other side effects were observed in the current study.

At baseline, there was no significant difference in general characteristics among groups. Nigella sativa supplementation significantly reduced anthropometric variables including weight, BMI, WC and HC in patients with Hashimoto’s thyroiditis (*P* < 0.05); while no significant change in placebo-treated group has been occurred (Table 1). Dietary energy and nutrient intakes before and after intervention are presented in Table 2. Energy and nutrient intakes were similar between groups before intervention and no significant change was observed after intervention. Serum TSH and anti-TPO concentrations reduced while serum T3 increased in Nigella sativa treated group (*P* < 0.05). Moreover, serum VEGF reduced significantly after 8 weeks of Nigella sativa supplementation (*P* = 0.02, Table 3). In stepwise multiple linear regression analysis when change in serum VEGF concentrations was entered as dependent variable and change in anthropometric variables and thyroid hormones as independent variables (Table 4) one model was obtained indicating change in WHR as predictor of change in VEGF concentrations. In similar procedure when change in serum Nesfatin-1 was entered as dependent variable, change in WHR, TSH and T3 were its predictors (*P* < 0.05).

**Table 1:** General characteristics and anthropometric variables in treatment groups before and after intervention

*N*	Nigella sativa	Placebo	*P*†
	*N* = 20	*N* = 20	
Age (years)	35.70 ± 8.18	33.95 ± 8.72	0.52
Levothyroxine (mcg/d)	119.85 ± 24.12	118.46 ± 22.12	0.91
Female [n (%)]	17 (85)	17 (85)	0.89
Weight (kg)			
Before	70.52 ± 12.27	69.63 ± 11.75	0.81
After	69.39 11.84	69.62 11.80	0.95
*P*‡	**0.004**	0.91	
BMI (kg/m2)			
Before	27.10 ± 4.63	25.93 ± 4.07	0.40
After	26.63 4.42	25.95 4.11	0.61
*P*‡	**0.002**	0.65	
Waist Circumference (cm)			
Before	88.56 ± 7.29	88.69 ± 7.41	0.95
After	87.72 ± 6.92	88.57 ± 7.35	0.71
*P*‡	**0.006**	0.17	
HC (cm)			
Before	102.85 ± 6.25	101.77 ± 6.84	0.61
After	101.56 ± 5.51	101.56 ± 7.02	0.99
*P*‡	**0.001**	0.08	
WHR			
Before	0.86 ± 0.052	0.87 ± 0.053	0.53
After	0.86 ± 0.05	0.87 ± 4.11	0.61
*P*‡	0.38	0.53	

*BMI* body mass index, *WC* waist circumference, *HC* hip circumference, *WHR* waist to hip ratio, †*P* values for ANOCOVA after adjustment for age, gender, duration of the disease and variable’s baseline value; ‡*P* values for paired *t*-test. Data are presented as mean ± SD or number (percent), the bolded *P* values are statistically significant

**Table 2:** Dietary intakes of energy and nutrients in treatment groups before and after intervention

*N*	Nigella sativa	Placebo	*P*†
	*N* = 20	*N* = 20	
Total calories (kcal/d)			
Before	2251.90 ± 349.58	2208.95 ± 327.80	0.69
After	2236.40 ± 248.27	2265.45 ± 270.73	0.72
*P*‡	0.77	0.32	
Carbohydrate (%)			
Before	57.11 ± 2.90	57.07 ± 3.78	0.97
After	57.24 ± 2.71	57.58 ± 3.32	0.72
*P*‡	0.26	0.67	
Protein (%)			
Before	15.73 ± 1.68	15.07 ± 1.29	0.17
After	15.77 ± 1.36	15.10 ± 1.81	0.19
*P*‡	0.94	0.94	
Fat (%)			
Before	27.34 ± 2.15	26.57 ± 2.32	0.28
After	26.56 ± 1.96	26.13 ± 2.48	0.55
*P*‡	0.51	0.51	
Vitamin E (mg/d)			
Before	2.98 ± 1.08	3.43 ± 1.48	0.36
After	2.89 ± 1.64	3.40 ± 1.19	0.28
*P*‡	0.80	0.96	
Vitamin C (mg/d)			
Before	79.75 ± 22.69	75.67 ± 17.24	0.52
After	28.37 ± 11.84	75.45 ± 15.36	0.59
*P*‡	0.77	0.91	

Data are presented as mean ± SD, †*P* values for ANOCOVA after adjustment for age, gender, duration of the disease and variable’s baseline value; ‡*P* values for paired t-test

**Table 3:** Metabolic parameters in treatment groups before and after intervention

*N*	Nigella sativa	Placebo	*P*†
	*N* = 20	*N* = 20	
TSH (mIU/l)			
Before	6.42 ± 3.86	8.14 ± 7.28	0.35
After	4.13 ± 2.35	8.27 ± 7.21	**0.02**
*P*‡	**0.03**	0.40	
T3 (mmol/l)			
Before	0.92 ± 0.27	1.18 ± 0.36	0.017
After	1.06 ± 0.34	1.16 ± 0.35	0.39
*P*‡	**0.008**	0.15	
T4 (mmol/l)			
Before	8.07 ± 2.56	7.97 ± 3.11	0.91
After	8.89 ± 1.43	7.63 ± 2.23	**0.04**
*P*‡	0.21	0.32	
Anti-TPO (IU/ml)			
Before	294.55 ± 210.05	278.10 ± 170.77	0.78
After	147.99 ± 158.33	274.30 ± 167.20	**0.01**
*P*‡	0.019	0.28	
Nesfatin-1 (ng/ml)			
Before	41.80 ± 28.33	25.86 ± 20.91	**0.049**
After	37.63 ± 5.91	26.75 ± 23.95	
*P*‡	0.34	0.69	
VEGF (ng/L)			
Before	3521.13 ± 395.95	2101.73 ± 339.29	0.17
After	2100.17 ± 36,082	2100.17 ± 360.82	0.25
*P*‡	**0.02**	0.99	

Data are presented as mean ± SD. † *P* values for ANOCOVA after adjustment for age, gender and baseline concentration of parameter; ‡*P* values for paired *t*-test. TSH, thyroid-stimulating hormone; *T3* triiodothyronine, *T4* thyroxine, *VEGF* vascular endothelial growth factor, the bolded *P* values are statistically significant

**Table 4:** Stepwise multivariate linear regression analysis in Nigella-sativa treated group with changes in VEGF and Nesfatin-1 as dependent variables and changes in anthropometric variables and thyroid hormones as dependent variables

	B	SE	β	t	P
Δ Nesfatin (as dependent variable)					
Δ WHR	387.54	183.92	0.24	2.10	**0.05**
Δ TSH	1.34	0.63	0.30	2.11	**0.05**
ΔT3	−59.11	14.49	−0.63	−4.07	**0.001**
Δ VEGF (as dependent variable)					
ΔWHR	35449.84	18234.88	0.31	1.94	**0.05**

*WHR* waist to hip ratio, *TSH* thyroid-stimulating hormone, *T3* triiodothyronine, *T4* thyroxine, *VEGF* vascular endothelial growth factor, *B* unstandardized coefficient, *SE* standard error, *β* standardized coefficient, *t* the student’s *t* distribution, *P* level of significance

## Discussion

In the current study we showed a meaningful impact of 8 weeks treatment with Nigella sativa on thyroid function, anthropometric features and serum VEGF concentrations in patients with Hashimoto’s thyroiditis. However changes in serum Nesfatin-1 concentrations were not significant. These findings were in accordance of findings of two animal studies; in one study by Khalawi AA [25] Nigella sativa oil improved hypothyroid status and decreased serum TSH concentrations in rats; in other animal study by Al-Asoom et al. [28] daily oral administration of 800 mg/kg Nigella sativa in male Wistar rats reduced serum thyroxine concentrations. However in our study, for the first time, we clearly demonstrated its beneficial role on improving thyroid function in human.

The seeds of Nigella sativa known as black seeds or black cumin have long been used in folk medicine in the middle and Far East as a traditional medicine for a wide range of disease including infections, obesity, hypertension and gastrointestinal problems [21]. Its most prominent constituent with well- known antioxidant, anti-inflammatory and anti-cancer properties is thyimoquinone [29]. Thyimoquinone has potential cytoprotective and anti-inflammatory effects; it has been reported that its anti-inflammatory effects are induced by up-regulated expression of heme-oxygenase-1 and suppression of the cyclooxygenase-2 (COX-2) expression in different cell lines [30]. Thyimoquinone also differentially modulated thyroid hormones and improved thyroid status in rats [31]. Therapeutic effects of Nigella sativa against hypothyroidism is mostly attributed to its antioxidant effects which have been proved in numerous studies [32–34]. It has also been suggested that Nigella sativa protects the hyperplasic changes of thyroid parenchyma in hypothyroid rats [25]. Accordingly, increment in T3 concentrations after treatment with Nigella sativa in the current study, has also been reported in the study by Ismail et al. [35] and the authors concluded that Nigella sativa could raise the lowered serum triiodothyronine concentration without changing the concentration of serum TSH because of its potential ability in repairing the thyroid gland and resynthesizing the thyroid hormone; therefore its therapeutic action could be in part due to antioxidant defense system. Accordingly, reduction of serum anti-TPO concentrations after treatment with Nigella sativa could be explained by its immunomodulatory effects approved previously by its protective roles against several autoimmune disease including type 1 diabetes mellitus and experimental autoimmune encephalomyelitis (EAE) [36, 37]. The possible underlying mechanisms of immunomodulatory effects of Nigella sativa are reduced synthesis of auto-antibodies, reduced innate and acquired immune cell markers and reduction in transforming growth factor (TGF)-β and interleukin (IL)-23 concentrations [36–38].

VEGF is minimally expressed in normal human thyroid cells [39]; however in pathological situations, enhanced TSH concentrations, is a potent stimulator of VEGF secretion [11]. It has been shown that VEGF and one of its receptors, Flt-1, are present in epithelial cells of the thyroid, and VEGF contributes to the regulation of development and function of thyroid epithelial cells [10]. Higher VEGF concentrations are associated with increased risk of recurrence and decreased disease-free survival in papillary thyroid cancer [40]. Strong expression of VEGF has been reported in thyroiditis and thyroid carcinomas [41]; therefore it is a critical cytokine in tumor angiogenesis and will be a potent target of diagnosis and therapy. In the current study, Nigella sativa had a strong impact in reducing VEGF concentrations in Hashimoto’s thyroiditis. It is mostly because of anti-angiogenic effects of Nigella sativa and its major bioactive compound, thyimoquinone, which has been proven previously in different cancer cell lines [42, 43]. Moreover, in the current study, change in WHR was a significant positive predictor of changes in serum VEGF in Nigella sativa treated group. In fact, VEGF is a multifunctional cytokine and its elevated concentration has been reported previously in several metabolic disorders including type 2 diabetes mellitus and polycystic ovary syndrome. A positive association between serum VEGF and its different genomic variants with the components of metabolic syndrome including central obesity and waist to hip ratio has also been previously reported [44, 45]. This relationship arise from this fact that adipocytes, specially white adipose tissue cells, produce VEGF which may act as an angiogenic and vascular survival factor for the omental vasculature and has paracrine or systemic endocrine actions, these might hypothetically impact on adipose expansion or the vascular comorbidities of obesity related disease [46]. In this context, it is interesting that Randeva et al. could reported a strong correlation of serum VEGF with waist-to-hip ratio in a considerable cohort of individuals (*χ* ^2^ = 17.42; *P* < 0.001) [47], a measure that, is suggested to be a better marker of subclinical arteriosclerosis and endothelial dysfunction [48] which are common clinical consequences of Hashimoto’s thyroiditis [49, 50].

Weight reducing effects of Nigella sativa has been observed in previous studies; Zaoui A [51] reported a significant reduction in body weight in rats after 6 weeks treatment with Nigella sativa fixed oil (*P* < 0.001). In other study 3 month supplementation with 1.5 g per day of powdered Nigella sativa in central obese men significantly reduced body weight [52]. One suggested mechanism is increasing mean rates of satiety and fullness [53]; although, we did not observe any change in dietary energy or nutrient intakes after intervention. Other possible mechanisms are reduced lipid absorption, increased energy expenditure, decreased pre-adipocyte differentiation and proliferation, or decreased lipogenesis and increased lipolysis [54]. The suggested underlying mechanisms of the effects Nigella sativa and its major ingredient thymoquinone’s on thyroid health and body weight are summarized in Fig. 2.

**Fig. 2:** The probable mechanisms of the effects of Nigella Sativa and its major ingredient Thymoquione on thyroid status and body weight. *TSH* thyroid stimulating hormone, *T3* triiodotyronin, *VEGF* vascular endotheilial growth factor

Hashimoto’s thyroiditis is more prevalent among females compared with males and women are up to 10 times more likely to develop the disease compared with men [55]. This strong female association remains unexplained although our hunch is that sex steroids have the critical role, as there is compelling evidence for such effects in animal models of many types of autoimmunity [56]. Other possible explanations include skewed X chromosome inactivation and fetal microchimerism [57]. Accordingly, the number of the female participants in the current study was more than men, but the gender distribution among two groups were equal. Therefore, the possible confounding effect of gender could be rule out. Moreover, the comparisons between all of the study parameters are adjusted for the possible confounding effects of age, gender and variable’s baseline values by ANCOVA.

In the current study serum Nesfatin-1 did not change after Nigella sativa supplementation in Hashimoto’s thyroiditis patients. The studies regarding the relationship between serum Nesfatin-1 concentrations and thyroid dysfunction are scarce and conflicting. One study in children demonstrated its reduced concentrations in children with untreated subclinical hypothyroidism [13]; while, other study by Sahin et al. [58] reported no difference in serum Nesfatin-1 concentrations in patients with hypothyroidism compared with healthy control group. Nesfatin-1 is colocalized with TRH and affects the membrane potential of TRH neurons in the paraventricular nucleus, which is known to be closely related to the regulation of thyroid function [15]. However we did not find any change in its concentrations after treatment with Nigella sativa. It could be due to relatively small sample size or treatment duration.

## Conclusions

We have demonstrated beneficial effects of Nigella sativa in improving thyroid status, reducing VEGF and body weight in patients with Hashimoto’s thyroiditis. Although no significant change in serum Nesfatin-1 concentrations has been observed, change in anthropometric variables and thyroid hormones were significant predictors of changes in serum Nesfatin-1 concentrations.

## Abbreviations

BMI: Body mass index
HC: Hip circumference
T3: Triiodotyronine
T4: Thyroxine
TG-Ab: Thyroglobulin antibody
TPO-Ab: Thyroid peroxidase antibody
TRH: Thyrotropin releasing hormone
TSH: Thyroid stimulating hormone
VEGF: Vascular endothelial growth factor
WC: Waist circumference
WHR: Waist to hip ratio
